The article "Resveratrol attenuates inflammation environment-induced nucleus pulposus cell senescence in vitro" was retracted in 2024. Reasons: duplicated images; compromised peer review; concerns about the authorship.

# Resveratrol attenuates inflammation environment-induced nucleus pulposus cell senescence *in vitro*

**DOI:** 10.1042/BSR20190126

**Published:** 2019-05-10

**Authors:** Xiaoming Li, Feixiang Lin, Yaohong Wu, Ning Liu, Jun Wang, Rongchun Chen, Zhijun Lu

**Affiliations:** Department of Spinal Surgery, Ganzhou People’s Hospital, Ganzhou 341000, Jiangxi Province, China

**Keywords:** cell senescence, intervertebral disc degeneration, nucleus pulposus, resveratrol

## Abstract

Intervertebral disc degeneration is a disease identified as an inflammation response-participated pathological process. As a classical cellular feature, disc cell senescence is reported to be closely related with disc cell senescence. Resveratrol has a protective role against inflammation in some cells. However, its biological effects on disc cells remain largely unclear. The present study was aimed to study the effects of resveratrol on disc nucleus pulposus (NP) cell senescence in an inflammation environment. Isolated NP cells were cultured in cultured medium with (control group) or without (inflammation group) inflammatory cytokine TNF-α and IL-1β for 14 days. Resveratrol was added along with the NP cells treated with inflammatory cytokines to investigate its effects. NP cell senescence was analyzed by senescence-associated β-Galactosidase (SA-β-Gal) staining, cell proliferation, G0/1 cell cycle arrest, telomerase activity, gene/protein expression of senescence markers (p16 and p53) and NP matrix biosynthesis. In addition, the intracellular reactive oxygen species (ROS) was also analyzed. Compared with the control group, inflammation group significantly increased SA-β-Gal activity and ROS content, decreased cell proliferation and telomerase activity, promoted G0/1 cell cycle arrest, up-regulated gene/protein expression of senescence markers (p16 and p53) and matrix catabolism enzymes (MMP-3, MMP-13 and ADAMTS-4), and down-regulated gene/protein expression of NP matrix macromolecules (aggrecan and collagen II). However, resveratrol partly reversed the effects of inflammatory cytokine on these cell senescence-associated parameters. Together, resveratrol was effective to suppress cell senescence in an inflammatory environment. The present study shows new knowledge on how to retard inflammation response-initiated disc degeneration.

## Introduction

Intervertebral disc degeneration (IDD)-caused pathological changes in the spine-associated tissues is a main reason for low back pain [1]. Current treatments for disc degeneration-caused spinal disease, either conservative therapy or surgical treatment, mainly aimed to alleviate pain syndrome, and these treatments cannot biologically retard or regenerate disc degeneration [2,3]. Until now, a biological strategy for disc degeneration is to be developed.

The central gelatinous nucleus pulposus (NP) plays an important role in retaining the spinal mechanical function [4]. It has been indicated that degenerative changes first occur in the NP region during disc degeneration [5,6]. Increasing evidence has indicated that cell senescence participates in the process of disc degeneration. Several previous studies have identified senescent cells in the disc tissue [6–9]. Moreover, cell senescence is positively related with the degree of disc degeneration [6,9]. Hence, inhibition of disc cell senescence may be an important point to retard disc degeneration.

Apart from disc cell senescence, inflammation response is another feature during disc degeneration. Previously, several studies have identified the existence of inflammatory cytokines (i.e. TNF-α and IL-1β) within the disc tissue, and demonstrated that these cytokines are increased in the degenerative disc tissue [10–13]. Some studies have showed that inflammatory cytokines induce cell senescence in some cell types, including endothelial progenitor cells and osteoarthritic osteoblasts [14,15]. Importantly, inflammatory cytokines often induces disc NP cell senescence in previous researches [16–18]. Therefore, we deduce that inflammation response-mediated disc NP cell senescence plays an important role in accelerating disc degeneration.

Resveratrol has some protective effects in different cell types, such as the anti-inflammatory and anti-aging [19–21]. Moreover, several studies have reported that resveratrol alleviates disc NP cell senescence under stimulation of certain pathological factors [22,23]. In the present study, we mainly aimed to investigate whether resveratrol is able to suppress inflammation environment-mediated NP cell senescence *in vitro*.

## Materials and methods

### Ethical statement

All animal experiments were processed according to a protocol approved by the Ethical Committee of Ganzhou People’s Hospital [SJTY(E) 2013-032].

### NP cell isolation and culture

Briefly, after NP tissue samples were separated from thoracolumbar spine (L5-T10) of Sprague–Dawley rats (6–8 weeks and 340–360 g weight), they were digested with 0.25% type I collagenase for 10–12 h at 37°C. Then, the isolated NP cells were plated in DMEM/F-12 medium with 10% fetal bovine serum (FBS, Gibco, U.S.A.) in a humidified atmosphere of 5% CO_2_. The second-generation NP cells were used for each experiment in the present study. The control NP cells were cultured in the baseline medium. The experiment NP cells were cultured in baseline medium with inflammatory cytokine TNF-α (20 ng/ml) and IL-1β (20 ng/ml) for 14 days. Resveratrol (100 μM) was added into the culture medium to investigate its effects.

### Intracellular reactive oxygen species content analysis

A reactive oxygen species assay kit purchased from a commercial company (Nanjing Jiancheng Bioengineering Institute, China) was used to measure the intracellular reactive oxygen species (ROS) content. Briefly, after NP cells were seeded in six-well cell culture plate and incubated with different test compounds for 14 days, they were incubated with the fluorescent probe DCFH-DA (10 μM) in a humidified atmosphere for 30 min at 37°C. Then, relative fluorescence units (RFU) was detected at an excitation/emission wavelength of 490/585 nm using an automatic microplate reader (Thermo, U.S.A.). ROS content was reflected by the RFU in the present study.

### Cell proliferation analysis

Cell proliferation was evaluated by CCK-8 assay. NP cells were seeded in the six-well cell culture plate (5 × 10^3^ cells/well) and incubated with different compounds. On days 1, 5 and 9, CCK-8 assay was performed according to the manufacturer’s instructions (Beyotime, China). Cell proliferation potency was reflected by the absorbance value at a wavelength of 450 nm.

### Senescence-associated β-Galactosidase staining

Briefly, NP cells were seeded in six-well cell culture plate and incubated with different test compounds for 14 days. Then, senescence-associated β-Galactosidase (SA-β-Gal) staining was performed using a Senescence β-Galactosidase Staining Kit according to the manufacturer’s instructions.

### Cell cycle analysis

Briefly, NP cells were incubated with different compounds for 14 days. At each time point, NP cell cycle was analyzed by flow cytometry. Briefly, after the cultured NP cells were fixed by cold ethanol overnight, they were stained with 50 μg/ml PI solution (Beyotime, China) for 30 min. Finally, cell fraction in each cell cycle phase (G0/G1, G2/M, S) was analyzed by a flow cytometry machine.

### Telomerase activity analysis

Telomerase activity was analyzed using a telomerase (TE) enzyme-linked immuno sorbent assay (ELISA) kit (Mlbio, China). Briefly, after NP cells were incubated with different compounds for 7 and 14 days, they were lysed using RIPA lysis buffer (Beyotime, China). Subsequently, the protein supernatant and the reaction buffer were mixed together to analysis telomerase activity according to the manufacturer’s instructions. Finally, after reading the absorbance values at 450 nm, telomerase activity (IU/L) of NP cells was calculated based on the standard curve that was created using the standard in the kit.

### Real-time PCR analysis

Briefly, after NP cells were cultured for 14 days, total RNA was extracted using TRIzol reagent (Invitrogen, U.S.A.) and synthesized into single-strand cDNA using PrimeScript™ II 1st Strand cDNA Synthesis Kit (TaKaRa, Japan). Subsequently, the cDNA templates were amplified by PCR using the specific primers (Table 1) and SYBR Green qPCR Mix (DONGSHENG BIOTECH, China). GAPDH was used as a reference gene and the relative gene expression was calculated by the method of 2^―△△*C*^_t_.

**Table 1:** Primers of target genes

Gene	Forward (5′–3′)	Reverse (5′–3′)
GAPDH	CCACCCAGAAGACTGTGGAT	CACATTGGGGGTAGGAACAC
Aggrecan	ATGGCATTGAGGACAGCGAA	GCTCGGTCAAAGTCCAGTGT
Collagen II	GCCAGGATGCCCGAAAATTAG	CCAGCCTTCTCGTCAAATCCT
p53	CCTTAAGATCCGTGGGCGT	GCTAGCAGTTTGGGCTTTCC
p16	TACCCCGATACAGGTGATGA	TACCGCAAATACCGCACGA
MMP-3	CAGTCCTGCTGTGGCTGTGTAC	AACCTCCATGCCAGCATCTTCTTC
MMP-13	AACCAAGATGTGGAGTGCCTGATG	CACATCAGACCAGACCTTGAAGGC
ADAMTS-4	CCGTTCCGCTCCTGTAACACTAAG	AGGTCGGTTCGGTGGTTGTAGG

### Immunocytochemistry analysis

After NP cells seeded on the coverslips were incubated with different test compounds for 14 days, they were washed with sterile phosphate buffer solution (PBS), followed by fixation with 4% paraformaldehyde for 15 min, permeation with 0.1% Triton X-100 (Beyotime, China) for 60 s and blocking with 5% bull serum albumin (BSA) for 25 min. Then, NP cells were incubated with the primary antibodies (aggrecan: Norvus, NB600-504; collagen II: Abcam, ab7778) at 4°C overnight and the horseradish peroxidase (HRP)-conjugated secondary antibodies for 1 h on the following day. After the positive staining was visualized using diaminobenzidine (DAB), NP cells were observed under a light microscope (Olympus EX51, Japan). The staining intensity was quantified using Image-Pro Plus software (Version 5.1, Media Cybernetics, Inc.).

### Western blot analysis

Briefly, after NP cells were incubated with different test compounds for 14 days, total protein was extracted using cell lysis buffer for Western and IP (Beyotime, China). Then, equal protein supernatant among these groups was separated by SDS/PAGE and transferred to the PVDF membrane. Thereafter, PVDF membranes were sequentially blocked with 5% BSA, incubated with primary antibodies (β-actin: Proteitech, 60008-1-Ig; p16: Novus, NBP2-37740; p53: Proteintch, 10442-1-AP. All diluted at 1:2000), and incubated with HRP-conjugated secondary antibodies (Cell Signaling Technology, 1:1000). Finally, protein bands on the PVDF membranes were visualized using ECL Plus (Amersham Pharmacia Biotech, Umea, Sweden) and densitometric analysis was performed using the Image J software (National Institutes of Health, U.S.A.).

### Statistical analysis

All numeric data expressed as mean ± S.D. in the present study were analyzed using the SPSS 17.0 software. The statistical difference between two groups was analyzed using a one-way analysis of variance (ANOVA). The *P*-value of less than 0.05 was considered statistically different.

## Results

### Intracellular ROS content analysis

Results showed that the intracellular ROS content in the inflammation group was obviously higher than that in the control group, whereas resveratrol partly decreased the intracellular ROS content of NP cells-treated with inflammatory cytokines (Figure 1).

**Figure 1:** Measurement of intracellular ROS content The intracellular ROS content in NP cells was measured by the fluorescent probe DCFH-DA. The numeric Data are expressed as mean ± S.D. (*n*=3). *: Indicates a statistical difference (*P*<0.05) between two groups.

### Cell proliferation

Results showed that the value of OD 450 in the inflammation group was lower than that in the control group, whereas resveratrol partly increased the value of OD 450 in the inflammation group on days of 1, 5 and 9 (Figure 2).

**Figure 2:** Cell proliferation analysis NP cell proliferation potency was evaluated by the CCK-8 assay. The numeric Data are expressed as mean ± S.D. (*n*=3). *: Indicates a statistical difference (*P*<0.05) between two groups.

### SA-β-Gal staining

Results showed that the SA-β-Gal staining-positive NP cells in the inflammation group was significantly higher than that in the control group. However, addition of resveratrol partly decreased SA-β-Gal staining-positive NP cells in the inflammation group (Figure 3).

**Figure 3:** Analysis of SA-β-Gal activity SA-β-Gal activity of NP cells was measured using a senescence β-Galactosidase staining kit. The numeric Data are expressed as mean ± S.D. (*n*=3). *: Indicates a statistical difference (*P*<0.05) between two groups.

### Cell cycle

Our results showed that NP cells in the inflammation group had a significantly increased fraction of the G0/G1 phase and a significantly decreased fraction of the S phase compared with the control group. Further analysis showed that resveratrol partly attenuated the effects of this inflammation environment on G0/G1 phase and S phase fraction in the inflammation group, which was reflected by the decreased fraction of the G0/G1 phase and a significantly increased fraction of the S phase after addition of resveratrol (Figure 4).

**Figure 4:** Cell cycle analysis NP cell cycle was evaluated by flow cytometry. Cell fraction in the G0/G1 phase, G2/M phase and S phase was calculated.

### Telomerase activity

Results showed that telomerase activity in the inflammation group was lower than that in the control group, whereas resveratrol partly increased the telomerase activity in the inflammation group (Figure 5).

**Figure 5:** Telomerase activity analysis Telomerase activity of NP cells was evaluated using a chemical kit. The numeric Data are expressed as mean ± S.D. (*n*=3). *: Indicates a statistical difference (*P*<0.05) between two groups.

### Expression of senescence markers

Results showed that gene expression of p16 and p53 in the inflammation group was significantly up-regulated compared with the control group, whereas resveratrol partly decreased their gene expression in the inflammation group (Figure 6A). Similarly, inflammation environment significantly increased protein expression of p16 and p53, whereas resveratrol partly decreased their protein expression in the inflammation group (Figure 6B).

**Figure 6:** Expression of senescence markers (**A**) Gene expression of p16 and p53 in NP cells was analyzed by real-time PCR analysis. (**B**) Protein expression of p16 and p53 in NP cells was analyzed by Western blot assay. The numeric Data are expressed as mean ± S.D. (*n*=3). *: Indicates a statistical difference (*P*<0.05) between two groups.

### Expression of matrix catabolism enzymes

Results showed that gene expression of catabolism enzymes (MMP-3, MMP-13 and ADAMTS-4) were all significantly up-regulated in the inflammation group compared with the control group, whereas resveratrol partly down-regulated their gene expression in the inflammation group (Figure 7).

**Figure 7:** Expression of matrix catabolism enzymes Gene expression of MMP-3, MMP-13 and ADAMTS-4 in NP cells was analyzed by real-time PCR analysis. The numeric Data are expressed as mean ± S.D. (*n*=3). *: Indicates a statistical difference (*P*<0.05) between two groups.

### Expression of matrix macromolecules

Results showed that inflammation environment significantly down-regulated gene expression of aggrecan and collagen II compared with the control group, whereas resveratrol partly increased their gene expression in the inflammation group (Figure 8A). In addition, inflammation environment significantly decreased protein deposition of aggrecan and collagen II, whereas resveratrol partly increased their protein deposition in the inflammation group (Figure 8B).

**Figure 8:** Expression of matrix macromolecules (**A**) Gene expression of aggrecan and collagen II in NP cells was analyzed by real-time PCR analysis. (**B**) Protein deposition of aggrecan and collagen II in NP cells was analyzed by Western blot assay. The numeric Data are expressed as mean ± S.D. (*n*=3). *: Indicates a statistical difference (*P*<0.05) between two groups.

## Discussion

IDD is a main contributor to low back pain [1]. Up to date, there is no biological treatment to regenerate or retard disc degeneration. Inflammation response and cellular senescence are two classical features during disc degeneration [5–13]. Furthermore, there is a positive relationship between inflammation response and disc cell senescence [16–18]. Therefore, inhibition of inflammation response-induced disc cell senescence may be helpful to retard disc degeneration.

In the present study, we evaluated NP cell senescence by using lots of parameters (i.e. SA-β-Gal activity, G0/1 cell cycle arrest, telomerase activity, gene/protein expression of senescence markers and matrix homeostatic phenotype) which are also used in previous studies. However, apart from these methods, there are also some other important parameters to evaluate cell senescence described in previous studies [24–26]. We investigated effects of resveratrol on disc NP cell senescence in an inflammation environment. Our results showed that inflammation environment significantly promoted NP cell senescence, whereas resveratrol partly suppressed NP cell senescence in the inflammation environment. The present study provides some theoretical basis for the efficacy of resveratrol in retarding inflammation environment-mediated disc degeneration.

Previous studies have showed that content of several inflammatory cytokines (i.e. TNF-α and IL-1β) are increased within the degenerative disc tissue [10–12]. In the present study, we used TNF-α and IL-1β to create an inflammation environment *in vitro* to imitate the inflammation microenvironment in the degenerative disc tissue. We found that this inflammation environment significantly inhibited NP cell proliferation, increased SA-β-Gal activity and G0/G1 cell cycle arrest of NP cells, decreased telomerase activity, up-regulated gene/protein expression of senescence markers (p16 and p53) and catabolism enzymes (MMP-3, MMP-13 and ADAMTS-4), whereas down-regulated gene/protein expression of NP matrix macromolecules (aggrecan and collagen II). All these results indicate that this inflammation environment promotes NP cell senescence *in vitro*. This confirms previous studies that inflammatory cytokine induces cellular senescence in disc cells and other cells [14–18]. In addition, the inflammatory factors (TNF-α and IL-1β) were maintained in the culture medium throughout the experiment in our study. So, this inflammation environment may exhibit a direct effect but not a long-term effect on NP cell senescence. Another issue needs to be noticed is that the proportion of senescent NP cells in the control group is relative high though there are some significant differences among these groups. In line with the present study, a previous study has indicated that NP cells exhibited features of senescence with increasing culture passages [27]. So, we speculate that certain culture conditions of *in vitro* cell culture or detection method may affect and even increase the number of senescent cells. However, these speculations need to be verified by further experiments.

Resveratrol shows an anti-inflammatory effects in some cells *in vitro* [28,29]. In disc cells, resveratrol also exhibits protective effects against certain pathological factors, such as inhibiting disc cell apoptosis, promoting disc matrix synthesis and inhibiting disc catabolism [23,30–32]. In the present study, we found that resveratrol partly stimulated NP cell proliferation, decreased SA-β-Gal activity and G0/G1 cell cycle arrest of NP cells, increased telomerase activity, down-regulated gene/protein expression of senescence markers (p16 and p53) and catabolism enzymes (MMP-3, MMP-13 and ADAMTS-4), whereas up-regulated gene/protein expression of NP matrix macromolecules (aggrecan and collagen II). These findings are consistent with previous reports about the protective effects of resveratrol and indicate that resveratrol is able to alleviate inflammation environment-induced disc NP cell senescence.

Additionally, previous studies have reported that inflammatory cytokines can provoke an oxidative stress that drives cells to premature senescence [33,34]. So, we also measured the intracellular ROS content among these groups. Results showed that ROS content in the inflammation group was obviously higher than that in the control group. In light of the aggravated cell senescence in the inflammation group, our results are in line with previous studies [33,34]. However, we also found that resveratrol partly decreased the intracellular ROS content of NP cells-treated with inflammatory cytokine, indicating that resveratrol is helpful to attenuate oxidative stress caused by an inflammation environment.

In conclusion, the present study first investigated the effects of resveratrol on NP cell senescence in an inflammation environment. Our results demonstrated that resveratrol attenuated NP cell senescence in an inflammation environment. The present study sheds a new light on the protective effects of resveratrol against inflammation response and shows new knowledge on how to retard inflammation response-initiated disc degeneration.

## Abbreviations

ADAMTS: a disintegrin and metalloproteinase with thrombospondin motifs
BSA: bull serum albumin
HRP: horseradish peroxidase
IDD: intervertebral disc degeneration
IL: interleukin
MMP: matrix metalloproteinase
NP: nucleus pulposus
RFU: relative fluorescence unit
ROS: reactive oxygen species
SA-β-Gal: senescence-associated β-Galactosidase
TNF: tumor necrosis factor
